# Effect of PCI Standardized Telephone Follow-Up Service Mode on Out-of-Hospital Complications, Rehospitalization Rate, and Quality of Life of Discharged Patients with Acute Coronary Syndrome after PCI

This article has been retracted.

**DOI:** 10.1155/2022/4319887

**Published:** 2022-07-21

**Authors:** Luyan Zhang, Yaling Tian, Hong Ren, Aihong Zhu, Li Dong, Xiuqin Wang, Xiaoyu Han

**Affiliations:** ^1^Patients Pay a Return Visit Department, The First Hospital of Qinhuangdao, Qinhuangdao 066000, China; ^2^Performance Management Section, The First Hospital of Qinhuangdao, Qinhuangdao 066000, China; ^3^CCU, The First Hospital of Qinhuangdao, Qinhuangdao 066000, China; ^4^Department of Geriatrics, The First Hospital of Qinhuangdao, Qinhuangdao 066000, China

## Abstract

**Objective:**

To explore the effect of percutaneous coronary intervention (PCI) standardized telephone follow-up service mode on out-of-hospital complications, rehospitalization rate, and life quality of discharged acute coronary syndrome (ACS) patients after PCI.

**Methods:**

From August 2020 to March 2022, 218 ACS patients who were discharged after PCI were included. The controls accepted routine nursing care, and the researches accepted PCI standardized telephone follow-up service mode. The nursing satisfaction, rehospitalization rate, out-of-hospital complication rate, blood lipid level, and life quality score were taken as the comparisons.

**Results:**

The nursing satisfaction of study group (100.00%) was significantly higher than that of control group (88.07%). The rehospitalization rate was dramatically lower in the study group (3/109; 2.75%) than in the control group (25/109; 22.94%) (*P* < 0.05). In addition, compared with the control group, the incidence of complications (acute myocardial infarction and angina pectoris) was significantly reduced in the study group outside the hospital (*P* < 0.05). The blood lipid levels of TCHO, TG, LDL-C, and HDL-C were lower in the study group than in the controls. Further, after nursing, the quality of life score of the two groups was both decreased with a higher quality of life score in the study group (*P* < 0.05).

**Conclusion:**

The application of PCI standardized telephone follow-up service mode in discharged patients with acute coronary syndrome after PCI can reduce out-of-hospital complications and rehospitalization rate and improve blood lipid level and life quality.

## 1. Introduction

Cardiovascular disease threatens human health in the world. The morbidity and mortality of cardiovascular disease have exceeded that of tumors. Coronary heart disease accounts for over 40% of cardiovascular disease-related deaths [1]. Acute coronary syndrome (ACS) is the most critical type of coronary heart disease. ACS is a complex acute myocardial ischemia syndrome. In terms of mechanism, coronary plaque fissures, erosion, and/or rupture allow highly thrombogenic substances in the plaque to enter the blood flow, causing platelets to adhere, activate, and aggregate on the damaged thrombus surface. Subsequently, different types of thrombosis appear and result in vascular stenosis or blockage, leading to corresponding myocardial ischemia or necrosis. Therefore, it is very important to quickly restore the blocked coronary blood flow after ACS to save the ischemic myocardium [2]. Emergency or elective percutaneous coronary intervention is the most common form of revascularization in patients with ACS [3]. The number of patients undergoing PCI surgery is increasing around the world. With the technical progress and the improvement of the number of PCI surgery, some problems begin to appear in front of people. In clinical work, we have found that readmission after PCI therapy is common [4]. Readmission after PCI can be regarded as an adverse event for patients. Patients may be readmitted because of complications related to PCI surgery or hospitalization. The underlying reasons can be divided into hospital factors, patient factors, previous disease factors, surgical factors, and drug-related factors [5–7]. Clinically, many explorations and attempts have been made to prevent patients from being readmitted due to various reasons, among which high-quality continuous care is considered to be effective in reducing the risk of readmission [8].

With the rapid development of the medical and nursing service market, telephone, as social software, has gradually attracted wide attention in various industries. Telephones will not be limited by time and space, and medical staff can use phones to communicate with patients in the form of language and text. If patients are not online, they can also establish good communication with patients by leaving messages [9]. In the continuous clinical practice, taking the patients' needs as the guidance and making full use of the telephone for the continuous nursing of the discharged patients have achieved certain results in improving reconsultation rate, compliance rate, satisfaction, and so on [10]. Therefore, it can be gradually promoted in a number of clinical professions [11]. For patients after PCI treatment, traditional continuous nursing often lacks real-time and nondiscontinuity. The standardized telephone follow-up service mode of PCI can push the relevant content by phone. Health education knowledge is released through text, pictures, language, and video messages, which makes the content of health education more intuitive and humanized [12, 13]. Patients and their families can make use of daily fragment time to read and watch repeatedly, which is conducive to the understanding of knowledge and the full mastery of skills [14, 15].

## 2. Materials and Methods

### 2.1. General Information

From August 2020 to March 2022, 218 patients with acute coronary syndrome who were discharged after PCI were picked. The subjects were randomized into two groups: control and study. The controls accepted routine nursing, and the study cases accepted PCI standardized telephone follow-up service mode. The age of control group was 50 to 76 years old (mean age 65.55 ± 3.43), consisting of 54 men and 55 women. The age of study group was 51 to 76 years (mean age 65.55 ± 3.42), including 51 men and 58 women. All of the patients gave their written consent.

Selection criteria are as follows: (1) patients who matched the diagnostic criteria of ACS [16]; (2) patients who received PCI operation during hospitalization; and (3) patients and family members voluntarily signed the informed consent form for this trial. Exclusion criteria are as follows: (1) patients have recently received thrombolysis or anticoagulation therapy; (2) patients were suffering from severe heart, liver, and other important organ diseases; (3) patients had allergic reactions and other adverse reactions to the drugs used in this study; and (4) patients with mental illness could not effectively cooperate with this follow-up treatment.

### 2.2. Methods

The control group received routine nursing interventions in the unit. The corresponding nurses are informed of follow-up at the time of discharge. The follow-up center develops specific follow-up questionnaires according to the disease, and each patient is given an individual follow-up plan. The follow-up contents are recorded, and the questionnaires are kept simultaneously in the form of a form to form a complete follow-up file. The medical staff and nursing staff of the department set up a WeChat group to regularly release health promotion pictures, videos, and notices to respond to the needs of discharged patients. The doctors and nurses in the department interact with patients in various ways such as live streaming, holding salons, workshops, and shake videos. The call center is responsible for regular patient follow-up reminders, appointment booking, health education, and question and answer sessions and provides a variety of out-of-hospital extended care.

The study group was given the PCI standardized telephone follow-up service model. The specific measures were as follows:

1. *The Platform Building*. The “patient follow-up service platform” is introduced, and common follow-up questionnaires are collected and submitted to the callback center. The health advisory team consists of three cardiologists, a deputy chief nurse in cardiology, and four senior return visitors. The headset telephones and computers are connected to the hospital intranet. The ACS patients after PCI treatment automatically access the follow-up service platform after the patient is discharged from hospital. Continuous nursing records or nursing return visit registration form are then established, and centralized telephone follow-up was conducted for each discharged patient after PCI treatment, mainly in the callback center
2. *Standardized Working Model*. The call center of the hospital inquires 7 aspects, including technical service issues, timely treatment, reasonable charge, therapy effect, honest practice, medical environment, and the overall situation of the hospital. For the patient requiring long-term treatment, patients with slow recovery and specific patients are asked about their recovery, and then, timely rehabilitation guidance should be given; the next follow-up of ACS patient with PCI is scheduled according to the disease template
3. *Standardized Service Process*. The service process standard clearly defines “What should be done every day and how?”. On this basis, weekly service process standard and monthly service process standards are formulated in strict accordance with the service requirements. The responsible person regularly supervises and inspects the service and discovery situation, so that problems can be corrected in time and the follow-up service can be improved continuously
4. *Friendly Language Exchange (Conduct and Language Specifications for Subsequent Telephone Service)*. Telephone etiquette, including the voice of the telephone service, has been standardized. Standardized operation specifications of voice service before, during, and after call are developed to make discharged ACS patients after PCI can feel the professionalism of callback to each other emotionally
5. *Timely Information Feedback*. Our hospital has developed a strict feedback mechanism for return visits. Each visitor is required to collect and organize relevant information in accordance with the regulations and procedures. The feedback information should be reported on the 10th and 25th of each month. If there is an urgent situation in discharged ACS patients with PCI, we need to communicate with the person in charge to solve the problem within 24 hours
6. *Digital Analysis and Statistics*. The data and indicators of discharged ACS patients after PCI, such as return visits workload, success rate of return visits, success rate of follow-up, and patient satisfaction, are digitally analyzed every month. The analysis results are summarized quarterly and discussed and summarized at a meeting. The quality of the return visit service is continuously improved on the basis of digital analysis

### 2.3. Observation Indicator

#### 2.3.1. Satisfaction

After consulting the literature and expert discussion, we designed patients' follow-up satisfaction [17]. There was a total of 10 items, including recorded patients' satisfaction with follow-up management mode, health education, medical and nursing service, and appointment registration process. It was divided into four dimensions: very satisfied, satisfied, general, and dissatisfied. Satisfaction rate = very satisfaction rate + satisfaction rate + general rate.

#### 2.3.2. Rehospitalization Rate

The rehospitalization rate of the two groups was calculated.

#### 2.3.3. Out of Hospital Complication

The incidence of out-of-hospital complications was calculated between the two groups.

#### 2.3.4. Blood Lipid Level

After admittance, total cholesterol, triglycerides, high-density lipoprotein cholesterol, and low-density lipoprotein cholesterol were all measured.

#### 2.3.5. Life Quality Scale

The life quality scale [18] consists of four subscales including physical, psychological, social, and health self-awareness. This evaluation has 29 items. The weight's Cronbach's coefficient ranges from 0.79 to 0.91. The level was graded from 1 to 5. The smaller the score, the greater the level of contentment.

### 2.4. Statistical Analysis

The database was established by the SPSS 20.0 software and described. Through *t*-test, chi-square test was used for counting data. The data of the same observation index before and after intervention were analyzed by repeated measurement variance. The ordered qualitative data were analyzed by rank sum test. The subjective cognitive score and objective index were analyzed by bivariate correlation analysis. The difference was statistically significant *P* < 0.05.

## 3. Results

### 3.1. The Nursing Satisfaction in the Both Groups

As shown in Figure 1, after comparing nursing satisfaction between the two groups, 90 cases were extremely pleased, 10 cases were satisfied, and 9 cases were common in the study group, and the satisfaction rate was 100%, while satisfaction rate in the control group was 88.07%, with 40 very pleased cases, 34 satisfied cases, 23 general cases, and 12 dissatisfied cases. Thus, the nursing satisfaction of study group was significantly higher than that of control group.

### 3.2. The Readmission Rate between the Two Groups

Compared with the rehospitalization rate in the control group (25/109; 22.94%), the rehospitalization rate in the study group (25/109; 22.94%) was dramatically lower (*P* < 0.05).

### 3.3. The Incidence of Complications outside the Hospital

The incidence of complications including acute myocardial infarction and angina pectoris was remarkably lower in the study group outside the hospital than in the control group (*P* < 0.05) (Figure 2).

### 3.4. The Blood Lipid Levels in the Two Groups

The blood lipid levels of TCHO, TG, LDL-C, and HDL-C were lower in the study group than in the controls (*P* < 0.05) (Table 1).

### 3.5. The Life Quality Scores between the Two Groups

As shown in Table 2, the scores of physiological function, psychological function, social function, and health self-cognition were both decreased in the two group after nursing with higher quality of life score in the study group (*P* < 0.05).

## 4. Discussion

Cardiovascular diseases are currently the leading cause of death among the elderly in industrialized countries, among which coronary artery diseases are the most common and lead to high mortality and high disability rates [19]. Among coronary artery diseases, acute coronary syndrome is a common clinical emergency with sudden onset and high mortality. It is one of the most important diseases leading to high mortality in the elderly in China [20]. PCI has gradually become one of the most important and effective means for the diagnosis and treatment of acute coronary syndrome. PCI can improve the degree of coronary stenosis and myocardial perfusion, significantly improve the ischemic myocardium, and then greatly reduce the mortality of acute coronary syndrome and improve the quality of life of patients [21]. PCI has become the mainstream of revascularization for patients with ACS in recent years because of its advantages such as less trauma, precise efficacy, controllable surgical complications, quick postoperative recovery, and short hospital stay [22, 23]. In addition to the influence of the patient's own condition and the operation itself, the lack of medical management and health services is also one of the important reasons. Based on this understanding, some studies have found that standardized and effective whole-course management of patients after PCI and the provision of high-quality extended nursing services effectively reduce the risk of readmission [24, 25].

After PCI treatment, patients with acute coronary syndrome will suffer from anxiety and depression and cognitive decline due to the gradual decline of physiological function, which can lead to decreased quality of life and self-management ability, increased rate of rehospitalization and mortality, and increased incidence of depression [26–28]. Thus, continuous nursing after discharge is particularly important. At present, continuous nursing mainly includes discharge guidance, family visits, telephone follow-up, and the establishment of continuous nursing centers. Although the establishment of continuous nursing center can communicate with patients face to face, the limited distance between nurses and patients, short time, and the lack of human resources result in the failure of continuous nursing, which seriously affects the recovery of patients and increases the risk of recurrence and death. In developed countries, telemedicine service through modern communication tools has become a new approach. With the popularity of the internet and smartphones in China, telephone follow-up visits have become the most common platform for doctor-patient communication. It costs nothing extra and does not take up much material and energy.

Routine telephone follow-up visits is a long-term medical support method in the past, which has a good intervention effect, but it is limited in time and space [29]. The inaccurate connection between patients and nurses at the time of the call may affect the efficiency of telephone follow-up. In addition, the object of telephone follow-up is relatively single, which often requires one-to-one contact between nurses and patients, resulting in a waste of time and resources, reduced work efficiency and lack of communication between patients [30]. The standardized PCI telephone follow-up service model is to provide telemedicine nursing service for patients through the social attributes of the telephone, thus providing timely and reliable nursing and rehabilitation knowledge for discharged patients. The service helps patients understand disease-related rehabilitation [31, 32]. Data show that the standardized PCI telephone follow-up service model integrates disease-related knowledge into resource in the form of pictures, text, and videos, providing a novel and interesting learning tool for patients [33–35]. PCI standardized telephone follow-up service model can fully reflect the concept of patient-centered nursing service, make patients feel care and attention all the time, improve the enthusiasm of patients to learn knowledge, and strengthen rehabilitation training [36]. In addition, the model has the advantages of simple operation, complete functions, many ages of users, and high user viscosity [37].

A previous study has reported that ACS patients who received nursing intervention of PCI had decreased hospital anxiety and depression scale but increased general self-efficacy scale scores compared with the control (patients who received routine nursing) [38]. Herein, we also found that nursing intervention was correlated with patients' anxiety, psychology, and self-efficacy. In addition, Liu et al. explained that anxiety, depression, sleep quality, incidence of adverse reactions, and self-management score of ACS patients in the experiment group (given evidence-based nursing) showed better results in comparison with the control group (given routine nursing care) after PCI [39]. In this study, we analyzed the application of PCI standardized telephone follow-up service mode in discharged patients with acute coronary syndrome after PCI for the first time. We found the nursing satisfaction of study group was significantly higher than that of the control group. The readmission rate of patients in the study group was lower than that of the control group. Moreover, the blood lipid levels of TCHO, TG, LDL-C, and HDL-C were lower in the study group than in the controls. Our data suggested that the application of the standardized telephone follow-up service model for PCI could improve prognosis. In addition, our results suggested that the standardized PCI telephone follow-up service model can effectively improve the knowledge of rehabilitation and facilitate acceptance of patients including middle-aged and elderly.

To sum up, the application of PCI standardized telephone follow-up service model in discharged patients with ACS after PCI can reduce the incidence of complications (acute myocardial infarction and angina pectoris) and rehospitalization rate, decrease the blood lipid levels of TCHO, TG, LDL-C, and HDL-C, and improve life quality, suggesting that this program is particularly useful and cost-effective in improving the prognosis of ACS patients after PCI.

## Figures and Tables

**Figure 1:** Comparison of nursing satisfaction between two groups.

**Figure 2:** Comparison of the incidence of out of hospital complications.

**Table 1:** Comparison of blood lipid levels between the two groups (*x̅*±*s*, mmol/).

Group	N	TCHO	TG	LDL-C	HDL-C
Control group	109	3.89 ± 0.42	2.94 ± 0.35	1.39 ± 0.44	1.99 ± 0.34
Research group	109	2.35 ± 0.41	2.01 ± 0.55	1.03 ± 0.31	1.41 ± 0.31
*t*		27.392	14.893	14.893	13.160
*P*		<0.01	<0.01	<0.01	<0.01

**Table 2:** The life quality scores between the two groups before treatment (*x̅*±*s*, points).

Group	*N*	Physiological function		Psychological function		Social function		Healthy self-cognition	
		Before nursing	After nursing	Before nursing	After nursing	Before nursing	After nursing	Before nursing	After nursing
Control group	109	15.84 ± 4.53	13.86 ± 2.95	16.44 ± 3.40	14.84 ± 4.12	18.61 ± 3.31	16.31 ± 2.44	15.31 ± 3.55	13.42 ± 1.65
Research group	109	15.42 ± 4.52	11.84 ± 2.96	16.42 ± 3.34	12.45 ± 1.33	18.66 ± 3.89	12.33 ± 3.55	15.32 ± 3.51	10.42 ± 2.52
*t*		0.685	5.046	0.043	5.763	0.102	9.646	0.020	10.398
*P*		>0.05	<0.01	>0.05	<0.01	>0.05	<0.01	>0.05	<0.01

## Data Availability

The datasets used and analyzed during the current study are available from the corresponding author upon reasonable request.
